The article "A review of plant leaf fungal diseases and its environment speciation" was retracted in 2026. Reason: compromised peer review.

# A review of plant leaf fungal diseases and its environment speciation

**DOI:** 10.1080/21655979.2019.1649520

**Published:** 2019-09-27

**Authors:** Archana Jain, Surendra Sarsaiya, Qin Wu, Yuanfu Lu, Jingshan Shi

**Affiliations:** a Key Laboratory of Basic Pharmacology and Joint International Research Laboratory of Ethnomedicine of Ministry of Education, Zunyi Medical University, Zunyi, Guizhou, China; b Bioresource Institute for Healthy Utilization, Zunyi Medical University, Zunyi, Guizhou, China

**Keywords:** Emergent diseases, environmental speciation, fungal pathogens, host plants, plants leaf disease

## Abstract

There is increasing difficulty in identifying new plant leaf diseases as a result of environmental change. There is a need to identify the factors influencing the emergence and the increasing incidences of these diseases. Here, we present emerging fungal plant leaf diseases and describe their environmental speciation. We considered the factors controlling for local adaptation associated with environmental speciation. We determined that the advent of emergent fungal leaf diseases is closely connected to environmental speciation. Fungal pathogens targeting the leaves may adversely affect the entire plant body. To mitigate the injury caused by these pathogens, it is necessary to be able to detect and identify them early in the infection process. In this way, their distribution, virulence, incidence, and severity could be attenuated.

## Introduction

Over 19,000 fungi are known to cause diseases in crop plants worldwide. They may remain dormant but alive on both living and dead plant tissues until conditions are conducive to their proliferation. Certain fungi may develop inside host plant tissues. Fungal spores are readily dispersed by wind, water, soil, insects, and other invertebrates. In this way, they may infest an entire crop [1]. In contrast, other fungi are, in fact, beneficial to the host plant and may support its growth and development. For example, mycorrhizae form a mutualistic relationship with host plant root systems. On the other hand, pathogenic fungi cause plant diseases such as anthracnose, leaf spot, rust, wilt, blight, coils, scab, gall, canker, damping-off, root rot, mildew, and dieback. Systemic foliar pathogens are major causes for yield and commercial crop losses and diminished crop quality [2]. The rapid identification of fungal disease by timely recognition of their symptoms is an effective management practice and may help control and prevent their spread and progress. Leaves with fungal lesions are photographed and compared with descriptions in databases uploaded on the internet. Fungal leaf diseases may be controlled if detected and correctly identified in a timely manner. Part of the crop disease management process includes assessing the negative impacts of the pathogens on crop yield [3].

The article "A review of plant leaf fungal diseases and its environment speciation" was retracted in 2026. Reason: compromised peer review.

**Figure 1.** Characteristics of environment speciation.

**Figure 2.** Disease control of plant leaf spot.

**Figure 3.** An overview of plant leaf diseases, its microbial and environmental interaction.

**Table 1.** Common leaf diseases caused via pathogenic fungi with its symptoms.

Year	Region	Plant	Causal agent	Disease	Symptoms	References
2004	Rajasthan and Sorghum, India	Maize	*Perenosclerospora sorghi*, *Perenosclerospora heteropogoni*	Downy mildew	Pale yellow to whitish discolorations on the leaf blade. Tassels may be deformed, and ears may be aborted.	[51]
2005	Western Turkey	Pear	*Erwinia amylovora*	Fire blight	First leafs turn yellow-brown and after that all are dying.	[52]
2007	New York	Carrot cultivars	*Alternaria dauci and Cercospora carotae*	Leaf blight	Brownish spotting on leaf.	[15]
2008	Belle Glade, USA	Celery	*Cercospora* *apii*Fres.	Early blight	Light-brown spots somewhat circular or slightly bony. Spots might be oily look with or with no nearby yellow coronas.	[53]
2009	Japan	Coronus Florida	*Anamorphic fungi*	Leaf blight	Dead and brown blotches on leafs.	[54]
2010	Egypt	Potato	*Phytophthora infestans*	Late blight	Pale green spots.	[55]
2011	France	Pear	*Erwinia amylovora*	Fire blight	First leafs turn yellow-brown and after that all are dying.	[56]
2011	Switzerland	Pea and apple	*Erwinia amylovora*	Fire blight	Red-brown to black streaking may be apparent in wood just under the bark.	[57]
2011	Parana Southern brazil	Soybean	Peronospora *menshurica*	Downy mildew	Upper (light green spots) and lower (greyish/beige downy tufts) on leaf surface.	[10]
2012	Germany	Apple	*Erwinia amylovora*	Fire blight	Red brown or black, may be outward in wood.	[21]
2012	Spain	Grapevine	*Plasmopara viticola*	Downy mildew	Lesions on leafs are angular, yellowish, sometimes oily, and located between the veins.	[58]
2013	Temanggung	Sengon	*Uromycladium tepperianum*	Gall rust	It starts with local swelling (tumefaction).	[59]
2013	North eastern India	*Capsicum assamicum*	*CercosporaFresen*	Leaf spot	Round or oblong spots occur; first water soaked and later turn tan with a dark marginal ring.	[60]
2013	France	Apple	*Erwinia amylovora*	Fire blight	The scorched appearance of plant leafs.	[61]
2014	Australasia and Southeast Asia	Grapevine	*P. montana*	Leaf rust	Angular brown spots on the topside of the leaf.	[62]
2015	USA	Tomato	*Phytophthora infestans*	Late blight	Pale green spots.	[63]
2015	Sanandaj, Iran	Chickpea	*Fusarium oxysporum*	Fusarium wilt	Grayish-green chlorosis, typically affecting lower leafs first and extending up the plant.	[64]
2015	Karnataka, Tamil Nadu, Andhra Pradesh, Kerala and Maharashtra, India	Tomato	*Alternaria solani*	Early blight	On leafs, circular lesions are produced. Inside these lesions turn dark, concentric rings could be seen.	[25]
2015	India	Pearl millet	*Sclerospora graminicola*	Downy mildew	Pale color, broad streaks spreading from bottom to top of leafs. Advancement of disease, the leaf streaks turn brown and leafs become shredded longitudinally.	[65]
2016	Egypt	Wheat	*Puccinia triticina Eriks*	Leaf rust	Rusty colored pustules erupting through on surface.	[66]
2016	Yunnan China	Pea	*Erysiphe pisi D.C.*	Powdery mildew	Brownish spots on leafs.	[67]
2016	Shandong, China	Apple	*Glomerella cingulata*	Leaf spot	Pale yellow, olive green and dark velvety spots.	[68]
2016	Sweden	Potato	*Oomycete Phytophthora infestans*	Late blight	Pale green spots.	[24]
2016	Hungary	Potato	*Phytophthora infestans*	Late blight	Pale green spots.	[69]
2016	Delhi, India	Maize	*Bipolaris maydis (Nisik)*	Leaf blight	In maize include tan, elongated lesions between veins with light brown to brown borders.	[70]
2016	Syngenta, Basel, Switzerland	Sweet Potato	*Alternaria solani*	Early blight	Leafs start to exhibit small irregular dark brown spots on the lowest part.	[71]
2017	Georgia, USA	Soybean	*Cercospora sojina*	Leaf spot	Dark brown centers with red or dark reddish margins.	[72]
2017	Mumbai, India	Tomato	*Fusarium oxysporum*	Fusarium wilt	Yellowing and wilting of lower leafs.	[73]
2017	Islamabad, Pakistan	Southern corn	*Cochliobolus heterostrophus*	Leaf blight	Southern corn include tan, elongated lesions between veins with light brown to brown borders.	[74]
2018	Tamilnadu	Groundnut	*Puccinia* *Arachidis Speg*	Leaf rust	Orange pustules on lower leaflet and rupture as masses of reddish brown urediniospores.	[13]
2018	Greece	Pea	*Erysiphe pisi DC*	Powdery mildew	Brownish spots on leafs.	[75]
2018	Peninsular Malaysia	Mango	*Fusarium*	Leaf spot	Gray to grayish brown spots with dark irregular margins.	[76]
2018	Chandigarh India	Eggplant	*Fusarium oxysporum*	Fusarium wilt	One side of leaf will wilt and stop expanding while the other side continues to develop.	[22]
2018	Northeastern Thailand	Rice	*Xanthomonas oryzae*	Leaf blight	Pale-green to gray-green than turn yellowish.	[29]
2018	Hawaii, Honolulu	Basil	*Peronospora belbahrii*	Downy mildew	Yellowish appearance, similar to a nutritional problem.	[27]
2019	Japan	Rose	*Phragmidium satoanum*	Leaf rust	Yellow black brown spots on both sides.	[23]
2019	Beijing china	Cucumber	*Oidium neolycopersici*	Powdery mildew	Appears dusty white yellow and gray coating on leaf surface.	[26]
2019	Canada	Strawberry	*Sphaerotheca macularis*	Powdery mildew	Grayish-white appearance on underside of leafs.	[76]
2019	Chandigarh	Grapevine	*Erysiphe* *necator*	Powdery mildew	Gray white powdery development on tissue.	[77]
2019	Guangzhou, China,	Peanut	*Puccinia* *Arachidis Speg*	Leaf spot	Circular dark brown spots surrounded by a yellow halo.	[78]
2019	Netherland	Potato	*Phytophthora infestans*	Late blight	Pale green spots.	[63]
2019	Shandong chins	Cucumber	*Trichoderma*	Fusarium wilt	Yellowing and wilting of lower leafs.	[20]
2019	USA	Cotton	*Fusarium* *oxysporum*	Fusarium wilt	Seem in the spring.	[79]
2019	Australia	Eucalyptus	*Teratosphaeria destructans*	Early blight	On leafs yellow brown patches and after some time they turn into dark color.	[80]
2019	Flakkebjerg, Denmark	Potato	*Alter aria solani*	Early blight	When leafs start turning to the small uneven dark brownish spots on top of the lower section.	[53]

The article "A review of plant leaf fungal diseases and its environment speciation" was retracted in 2026. Reason: compromised peer review.

**Table 2.** Host-specific plant leaf disease treatment along with prevention approaches.

Disease	Host plant	Treatment	Prevention
Powdery Mildew	Pea, cucumber, strawberry, and grapevine	Treated with sulfur; apply chemicals on vegetables once the disease signs appear; Eradicate the diseased crops to mitigate the pathogen spread.	Pathogen endures in dry and cool conditions; avoid such conditions to mitigate the pathogen.
Fusarium wilt	Cucumber, cotton, eggplant, chickpea, tomato	Best approach to control disease by using disease-free seedlings or plant-certified seed; Kill the pathogens by applying fungicides, for example Cap tan, Terraclor, Mycostop, and Thiram; safely defend the crops against wilt disease cause over fusarium.	Harmful microbes are prevented by maintaining the garden temperature lower; disinfect and clean farming tools before using them.
Fire blight	Pear & apple	Avoid heavy or low application of fertilizer, both encourage the growth. Avoid planting nearby to wild crops. Once fire blight is appeared, prune off diseased branches one-foot underneath the diseased segments and prevent by burning them to reduce further infection.	Never apply high nitrogen fertilizer
Leaf spot	Peanut, mango apple, soybean and capsicum	Not use overhead water; Decrease humidity among plants by providing adequate space among plants and by pruning lesser branches; Use mulch below trees.	Remove and dispose of spotted leafs on plants that have fallen. Apply sulfur sprays with copper base fungicides in a week after first disease sign to stop its spread from sprouts. Safely manage utmost fungal as well as bacterial disease.
Leaf rust	Sengon, grapevine, wheat, ground& rose	The best way to control white rust is to practice crop rotation. Concerning treatment, try appropriate fungicide to destroy the microbes.	Prevent Albugo through disposing crop separate before planting the crop.
Downy mildew	Basil, soybean, pearl millet, grapevine & maize	Control downy mildew through uprooting the diseased crop along with burn; treat it through forestry-al fungicide.	Prevent the pathogen by avoiding wet and cold conditions; prevent excess overhead irrigation and watering.
Leaf blight	Maize, rice, Cornus florida, corn, carrot	In summer, eliminate limbs, cutting well external infected area and dispose.	Avoid excess of feed along with severe pruning.
Early blight	Eucalyptus, potato, cerely and tomato	Spread copper base fungicides early sign before 2 weeks of disease; cover equally the tops and undersides leafs.	Stake or prune plants to expand air flow and decrease fungal complications; Disinfect pruning shears after each cut; Keep the clean soil under plants; Trickle irrigation and downpour hoses are useful to support keep the foliage. Burn infected plant portions.
Late blight	Potato and Tomato	Remove diseased parts prior to planting and space plants far sufficient apart to permit for sufficiently of air passage; Watering in early morning time, to give plants period to dry ready during the day-evade overhead irrigation.	Keep eyes on the plants for understand the disease complications at early stage; Protection by spraying plants with fungicides which help to prevent late blight infection.

[62,63,67,81–83]

Human populations rely heavily upon consistent and stable agricultural production. Foliar fungal diseases may pose serious threats to food security. Various disease recognition techniques are required for the rapid detection of leaf diseases in the early phases of plant growth and fungal infection [4]. The current approach for leaf disease recognition is based on the identification and detection of fungal pathogens by comparison with databases from national or regional biological information systems. However, this approach is not fully reliable. Over the past two decades, leaf diseases have been investigated using visible array images. Nevertheless, the methodology to date is imperfect and tends to rely upon idealized disease models and scenarios [5]. Although the focus here is the accurate identification of foliar fungal diseases, environmental speciation may render this task difficult and challenging. Details of research methodology including the networks and software packages used were omitted as they are beyond the scope of this article. This review article surveys emerging fungal leaf diseases, addresses the effects of environmental speciation, and discusses the complications associated with foliar fungal disease recognition.

The article "A review of plant leaf fungal diseases and its environment speciation" was retracted in 2026. Reason: compromised peer review.

## Significance and characteristics of emerging foliar fungal diseases

In environmental speciation, barriers impede the flux of genetic material between populations, but environmental factors induce mutations that result in new species. In optional speciation, the growths of pathogens are dependent on the environment basis at the earlier stage. The human actions are contributed toward the variations of bio network. . There is growing evidence that these fluctuations play major roles in determining the establishment of microbial pathogens in plants [6]. In this regard, many researchers have concentrated on the increasing incidence of fungal leaf diseases on the host owing to its significance with a consequence of the profusion of recognized cases. The significances of different fungal illnesses on the host are important for agricultural yield under the natural environment. However, this theoretical structure does not account for adaptation or differences among pathogens despite evidence that the contamination of a new plant could increase the incidence of developing diseases [7].

Information about fungal leaf diseases is required for the study of well-known views of environment speciation. It can enhance the host plant's  physiology and the growth due to its environmental speciation interaction with pathogens. There are several indications that plant pathogens may undergo rapid environmental speciation via changes in the host itself. Elucidation of the connections among emergent diseases and environmental speciation will help in the development of more realistic models and simulations that integrate the characteristics of the fungal pathogen and new experimental methods to study them. These incidences are responsible for the growth of fungal leaf illnesses [8].

### Characteristics of environmental speciation

Pathogen virulence may be determined by a single diallelic loci in the pathogen and the host. Host resistance may be identified when the host transports a resistant allele and the pathogen carries an avirulent allele. The allelic mixtures facilitate contagion as the host does not transport the unaffected allele, or while the pathogen carries the ‘deadly’ allele that escapes host recognition. Pathogen alleles are called as virulent strain. It can denoted as virulence for the qualitative capacity of the host genotype(Figure 1) [9].

Plants could change speciation through concentration on a fresh mass. Obligate biotope is a pathogenic living organism that gains resources from the host. Though, lots of mysterious varieties have been discovered inside morphological varieties through utilizing the hereditary concordance of phylogenetic strain for reorganization measures. These strain criterions are used for the phylogenetic concordance of many nonlinked genes. The phylogenetic strain reorganization decisive factor has proven considerably useful for fungi as it is frequently more discerning than other criteria and is also more convenient to use. We regard the whole fungi capable of reproduction. Moreover, the cross-strain communication of pathogen can be stored in the organization of new tissue [10].

The article "A review of plant leaf fungal diseases and its environment speciation" was retracted in 2026. Reason: compromised peer review.

### Characteristics of fungal pathogens of plant leaves promoting environmental speciation

Some history characteristics of fungal pathogens are favorable to environment speciation as they reduce the constraint for harmful speciation. We detail these features below and speculate their significances for the probability of environment changes. The number of spores is a particularly important determiner determination of alteration input for individuals. Pathogenic fungi can generate thousands of microspores in lesions and lead to considerably increased propagation in similar hosts that could give way to split the diseases [11]. Furthermore, high spore numbers permit the rapid generation of gene differences via mutation. Original variety of resistance gene can confer the full confrontation inside for only some months [12].

Such quick development could arise uniformly for growing pathogens and could be identical for lower inherited multiplicity. If the progeny is lower, the selection of plant could be vital intended for the progeny through the superlative probable inherited with ecological circumstantial. This ‘magical trait’ state is a single trait and is mainly favorable for environmental speciation. In theoretical models, the restriction on gene flow is the reduced viability of emigrants. With a very robust choice, it can totally avoid the impartial genetic transformation. Several studies have provided an experimental evidence for the generalization of a mechanism in fungal host pathogens [13,14].

## Emerging plant leaf fungal diseases

Pathogenic fungi are responsible for ≤30% of all crop diseases. Epidemics caused by a fungal pathogen and the changes they cause to ecosystems must be reported. Well-documented outbreaks of *Cryphonectria parasitica* on chestnut trees have resulted in nearly 100% defoliation. Another more recent blight was caused by *Phytophthora cinnamomic* which is responsible for root rot or dieback in numerous crops. Devastating fungal diseases may affect multiple host plant species and indirectly involve beetles, birds, and other animals. *Phytophthora infestans* was responsible for potato blight in Ireland. Fungal blast has infested wheat in Brazil since the 1980s and has advanced toward other South American nations. The fungal pathogen *Puccinia graminis* has case wheat stem rust [15,16]. Following are descriptions of various important fungal plant pathogens (Table 1).

The article "A review of plant leaf fungal diseases and its environment speciation" was retracted in 2026. Reason: compromised peer review.

### Fungal leaf spot

Plants cause an effect on the main production with economic losses of farming crop. It can be improved by identifying the leaf sicknesses inside the early-on leaf with disease identity. It can be capable of making easy the recognition of the diseases by a suitable strategy. Here, the current processes for an earlier finding of leaf diseases inside the host are based on the numerous significant structures examined from its leaf descriptions. Leaf spots become visible about 1 week after they first appear. They are white to grayish-white on the edges and enclosed by reddish-brown, brownish, or yellowish margins [17]. They are first observed on the adaxial leaf surfaces and then become apparent on the abaxial leaf surface as well. Ultimately, they perforate the lamina. These holes may vary in diameter and outline shape or may be identical to the initial spots. In general, it is the newer (younger) leaves that first present with fungal lesions. There may be a few small spots that enlarge over time. Others may coalesce or merge into blotches [18].

The main control measure for fungal leaf spot diseases is to keep the foliage as dry as possible. Plants in greenhouses should not be placed directly under overhead watering. Irrigation should only be applied to the roots in the potting media. The spores of the causative fungi are dispersed by water droplets, personnel working with wet infected plants, and mites and insects. The spores may germinate in water or inside the natural leaf openings (hydathodes, lenticels, stomata, etc.) [19].

### Leaf blight

In leaf blight diseases, the tips and margins turn yellow (chlorotic). Necrosis ensues, spreads, and forms dark-brown patches variable in size. As tissue death progresses, eventually the entire lamina dies. Older leaves are generally more susceptible to this disease [20].

### Fire blight

*Erwinia amylovora* is a bacterial pathogen causing fire blight on pear, apple, cotoneaster, and other Rosaceae. Numerous genes associated with the pathogenesis of *E. amylovora* and fire blight have already been characterized. The bacteria penetrate the host plant via its natural openings such as nectarthodes as well as wounds on the damp aerial organs. Unlike certain plant fungal pathogens, *E. amylovora* causes a localized necrosis and does not radiate to or colonize adjacent plant tissues [21].

### Fusarium wilt

Fusarium wilt is a serious vascular wilt disease in crop plants. It is caused by *Fusarium oxysporum* which may be morphologically indistinguishable from nonpathogenic strains. The spores spread through soil, plant debris, and seeds and are difficult to eliminate from infested fields and plants. Fusarium wilt attacks potato, tomato, and other *Solaneceae*. The leaves and possibly the stems of infected plants lose turgidity, turn light green to greenish-yellow to brown, and finally collapse and die. Biological controls have generally been effective in the management of this disease. Plant resistance proteins also confer protection by directly or indirectly reacting with fungal pathogen virulence proteins [22].

The article "A review of plant leaf fungal diseases and its environment speciation" was retracted in 2026. Reason: compromised peer review.

### Leaf rust

There are >4,000 known species of leaf rust. They infest beans, tomatoes, roses, and other crops. The lesions first appear as white, slightly raised spots on the lower epidermis of the lower (older) leaves of mature plants. Over time, the lesions are covered with red-orange spore masses. Later, pustules form and turn yellow-green and eventually black. Severe infestations cause foliar chlorosis, deformation, and eventual abscission [23].

### Late blight

Late blight is a systemic infection caused by the fungus *Phytopthora infestans*. It often occurs during plant growth and development and may appear after flowering. It starts with the oldest leaves and manifests as green and gray spots on the leaf surfaces. As the disease progresses, the spots darken and white mycelial masses form on the lower leaf surfaces. Finally, the entire plant is infected. This pathogen does not overwinter in the soil or garden litter. It is introduced via contaminated tubers, transplants, and seeds [24].

### Early blight

This disease commonly occurs on potato and tomato. The causative agent is *Alternaria solani*. Lesions first appear on lower epidermis of older leaves. They appear as small brown spots consisting of concentric rings arranged in a bullseye pattern. As the disease progresses, the lesions spread and cause the leaves to turn yellow, wither, and die. Finally, the infection may also radiate to other parts of the plant. The pathogen overwinters in contaminated plant tissue and is transmitted by rain, irrigation, insects, and gardening tools. It is also transmitted by infested potato tubers and tomato seeds. Despite its name, early blight may occur at any time during the plant growth period. It often attacks malnourished or distressed plants [25].

### Powdery mildew

This disease is caused by a wide variety of fungal pathogens with limited host ranges. It first appears early in the plant growth period. Powdery mildew starts on budding leaves and forms blisters causing them to curl upwards and expose their lower epidermis. The upper surfaces of the infected leaves eventually become covered with a fine white to grayish powdery mycelial mass. Flower buds infested with powdery mildew may be inhibited from opening. Eventually, the leaves may become necrotic and abscise. The pathogen preferentially infests younger leaves with high moisture content. Mature leaves are less commonly infected [26].

The article "A review of plant leaf fungal diseases and its environment speciation" was retracted in 2026. Reason: compromised peer review.

### Downy mildew

Downy mildew (*Plasmopara viticola*) affects numerous plant species. It manifests as yellow-to-white patches on the upper surfaces of mature leaves. The fungus forms downy mycelial masses that appear after rain and heavy dew and then rapidly regress after sun exposure resumes. Infected leaves turn brown and papery and may abscise despite adequate internal moisture. Downy mildew is cold tolerant and the pathogen resides in the plants and the soil. The spores are transmitted by insects, wind, rain, and gardening tools [27].

### Appearance of plant leaf fungal diseases in host alteration speciation

Emergent diseases could arise from a rapid increase in virulence owing to geographic variation in an earlier overlooked pathogen, followed by infection of a fresh host, which is the most common cause of the development of new fungal diseases. Infection of new plants could be an outcome from an association, plant array enlargement, or host alteration. A lot of attention has been dedicated toward the extrinsic features that facilitate interaction between a pathogen and a fresh host, for example, changes in surrounding climatic conditions owing to global trade [28]. Even though, the pathogens could be premodified from contamination with communication on an original kind of tissue. It is mainly dominant illness appearance in the form of pathogen [19].

The existing development concepts are expressed as the revision on the new plant leaf. The movement of inherited genes could be terminated partially or completely. These are building the development of propagate the separation of growing diseases . Differentiations are found when observed for the variation inside C. parasitic. Another historic case of disease appearance is occurred due to the environmental speciation via host shifts. These factors are generally confined the prospect of speciation [29]. The current concept of environment speciation might be accustomed to better understand the to better understand the aspects or opinion inside natural science as well as development encouraging the revision of pathogens toward a novel plant leaf. The horizontal genes can move through inter-specific hybridization.  It has been revealed that the pathogens can give the appearance of fungal disease on the new plant leaf, but as revision is generally the outcomes of assortment with obtainable gene’s alternatives or new changes inside fungal inhabitants [21,30].

The article "A review of plant leaf fungal diseases and its environment speciation" was retracted in 2026. Reason: compromised peer review.

## Inferences of concern regarding growing fungal diseases and environment speciation

Know that the increase in illnesses can be caused through the fungal host pathogens frequently. The abundant characters of fungal host pathogens can cause under favorable condition of environment speciation. This will have better insights into modern tools used for investigation of illness with the multiplicity of fungi. Moreover, this has implications for our understanding of how disease development affects variation, in addition to manipulative well-organized sustainable management plans. First, if changes in the host alone might be enough for speciation, then interfertility, one of the major’s criterion, generally applies for the delimiting varieties. Inter-fertility might be retained along gene flow between the host pathogen's types. On the other hand, the plant leaf variation might be a well-organized barrier to facilitate speciation via plant alterations. It is indicated that two dissimilar pathogenic variabilities can be measured in the same manner as in other studies [31]. This could allow for improvement of regulatory processes that determine the specificities of every class, for example, definite fungicide resistance. Furthermore, host adaptation only could be allowed for identical quick speciation through a host shift, so the rapid development of disease indicators would be desirable to identify the strains.

Additionally, it is significant toward linkage of emergent diseases with environment speciation in the path of measure if novel diseases owe toward spread, host variety growth, or host alteration speciation. These changed circumstances are affected the control measures to be taken. Furthermore, the changing aspects and disease development will be dissimilar if the pathogens are modified toward an only against numerous plants [32,33]. At last, if host variation is adequately intended for speciation on an original plant by host changes, then the illness appearance could be reasonably spread more steadily. Furthermore, samples for the development of fungal pathogen characteristics can acquire in the account for the specificity of the pathogen’s growth. Furthermore, the disease management strategy is considered for which the pathogens are caused the main grave symptoms like plants fungal pathogen’s interact inside their hosts and cause disease appearance on new tissues [34].

## Recent approaches and research trends for disease management

### Single and static management strategies

The control of plant leaf pathogens is difficult partly because of their progressive changing behavior and development associated with high genetic variation and rapid growth periods, which allow them to overcome the recently highest effectual disease (Table 2 and Figure 2). It is described that the proportions of augmented pesticide are used to indicate the reduced competence with economic comeback of used pesticides toward plant disease. Generally, pesticides could be used in a regime that regulates the timing, frequency, and amount of application, independent of the specific resistance status, and ecological environments. The safe and immobile approach of pesticide utilization does not only decrease the effectiveness of the management and increase the expenses, but also has adverse environmental consequences, such as toxicity toward livestock [11,35].

The article "A review of plant leaf fungal diseases and its environment speciation" was retracted in 2026. Reason: compromised peer review.

### Gray box of plant disease plague mechanisms

Rapid and prompt crop disease prediction, recognition, and analysis are essential. Molecular methods are currently being used to characterize and analyze plant pathogenesis. Despite the availability of these techniques, they are not universally applied here as the agricultural industry may still rely upon agronomists with traditional knowledge using conventional research methods. Accurate and effective crop disease assessment requires an in-depth understanding of the pathogenesis, pathogen–environment intercommunication, and influential biotic and abiotic factors involved. In view of these complexities, with a few notable exceptions, accurate, timely crop disease forecasting remains imperfect [34].

### Financial examination of host leaf disease management

Optimistic externalities can show the profits by the disease management within the farms for reduce the possible pathogens. Presently, these optimistic externalities are not listed in the commercial investigation of host disease management [36]. Growers must account for expenses incurred from pesticide application but not for those connected to residue elimination or site remediation. As growers are only compensated for their crop disease management costs, they select strategies that generate the highest immediate returns possibly while discounting the potential negative ecological impacts of the pesticide deployments. Certain highly effective disease management strategies are in current use without adequate regard for their long-term adverse environmental effects [37].

### Prospects of plant leaf disease management

Sustainable leaf disease management is needed for the multidimensional concern, includes social, financial side with environmental science. The host leaf disease management approach could be useful to explore not only single traits but also to shield the natural atmosphere. Future investigations in biological plant leaf disease management must focus on:

1. global and evolutionary outlines of leaf disease under changing environmental conditions and production demands;
2. ecological impacts on crop yield and pathogen resistance;
3. social and financial evaluation of leaf disease outbreaks and their management; and
4. technological development for the combined management of major crop diseases and environmental protection [38].
5. assurance of food security, safety, quality, and variety as human populations grow and living standards improve;
6. declining crop production as a result of competitive use and overuse of farmlands and possible soil nutrient depletion;

Future plant disease management should aim to improve food safety for the growing population while simultaneously preserving ecosystem integrity by reducing dependence on the most commonly used resources. The leaf organizations are the chief component for the normal adjustment of confrontation, removal and remediation strategy. It is directed through characters of host–pathogen relations by evolutionary bionetwork values to make ecological (biotic and abiotic) circumstances positive for host development [39,40].

The article "A review of plant leaf fungal diseases and its environment speciation" was retracted in 2026. Reason: compromised peer review.

Fungal diseases intimidate financially prominent plants leading toward important financial losses universal. Fungal pathogens can damage the food production for worldwide food demand. The significance of emergent fungal plant leaf pathogens must be assessed with progressive, rapid, and accurate disease recognition tools. Unfortunately, many currently available technologies and strategies are inadequate in these respects. They may be cost- and labor-intensive, slow, inefficient, and complex. Molecular and immunological tools generate highly informative data but require special equipment and personnel trained and qualified to use them. Novel methods and approaches must be able to deliver accurate results rapidly and identify plant leaf diseases early in their progression. Biosensors help improve the disease recognition capabilities of diagnostic tools. Several of them have been described in the literature [41,42]. Their efficacy has been tested in artificial field trials under controlled conditions, but they still require evaluation on imminent disease outbreaks under natural and real crop field conditions.

Biosensors may be designed and programmed for high throughput using nanomaterials, nanofabrication technology, and DNA sequencing [37]. The ongoing emergence of microbial plant pathogens could result in major financial and yield losses in agriculture. Bacterial leaf diseases are treated with copper-based compounds and antibiotics. However, pathogens may acquire resistance to them and they may have negative ecological impacts. Moreover, the improvement of antibiotics has been helpful for the ability of a well-organized crop shield. This condition is driving the investigators toward travel around novel and non-conventional methods [43]. Antimicrobial peptides have attracted attention as potential biological controls for plant leaf diseases. These compounds have amphipathic structures that interact with the anionic phospholipids of fungal membrane and cause their disruption [44].

The article "A review of plant leaf fungal diseases and its environment speciation" was retracted in 2026. Reason: compromised peer review.

## Challenges and upcoming outlooks

Accurate diagnostic methods that can be used *in situ* to detect plant disease must be developed, tested, and perfected in the near future. New fungal leaf disease identification technologies designed for field use may incorporate DNA sequencing. However, sampling and the use of this technology in the form of transportable biosensors may be logistically challenging. Moreover, onsite DNA sequencing expertise may be difficult to acquire as plant leaves have large and complex genomes [45]. For data mining and analysis, high-throughput computational biology and informatics will be essential. At this time, there are no initiatives being undertaken to improve transportable DNA sequencing biosensors that effectively identify fungal plant pathogens. Sequencing with microfluidic devices will facilitate the recognition of numerous fungal plant pathogens in the future. The application of biosensors in fungal diagnostics will enable the development of miniaturized, cost-effective, accurate, simple, and rapid apparatus that can readily be used on-site and in the field even by untrained personnel [46].

Extensive investigation is necessary for additional manipulation of biological approaches and viable applications (Figure 3). However, recognition of molecular markers connected through disease-resistant key genes and quantitative trait loci display the possible application of marker-aided choice in plant disease resistance [47]. PCR and flow cytometry may eventually be implemented in the genetic recognition of existing pathogens and the identification of emergent ones [48]. Genetic investigations could detect sources of pathogen and host resistance in diseases such as powdery mildew. Biological control in the form of seed dressing has been evaluated against root rot fungal pathogens such as *Trichoderma* [47]. RNA sequencing and double-stranded RNA may be deployed to recognize exclusively fungal genetic biomarkers [49].

Management of foliar fungal diseases involves both physical and cultivation approaches including the manipulation of plant resistance and the use of synthetic fungicides, bioproducts such as natural plant extracts, and defense activators or biostimulants. The application of thermography for disease evaluation is limited and flawed as it is highly sensitive to fluctuations in ambient environmental conditions [47,48]. Another option is the examination of individual targeted molecules. However, it is not generally accepted as it discloses only a fraction of the entire chemical profile. Analysis of untargeted volatile organic compounds provides a broader view of the host biochemical organization. This technique may be applied even when highly dissimilar volatile organic compounds must be immediately and simultaneously detected and quantified. Remote-sensing methods may also prove useful in fungal crop disease monitoring [50].

The article "A review of plant leaf fungal diseases and its environment speciation" was retracted in 2026. Reason: compromised peer review.

## Conclusions

Integration of biosensing mechanisms and DNA sequencing technologies will enhance the accuracy of fungal crop disease detection. Here, we reviewed several major plant foliar fungal pathogens and the factors that induce environmental speciation and host shifts in them. Fungal leaf diseases are responsible for major yield losses in commercially important crops worldwide. In addition to evaluating the agricultural significance of fungal leaf diseases, it is necessary to develop tools that enable the rapid recognition of these disease tools. One possible approach is the identification of environmental speciation in these pathogens.

## Highlights

- This review explored the factors that controlled the emergence of leaf fungal diseases;
- Recent approaches and research trends are helpful to leaf disease management;
- Economic analysis played an important role in planning of plant disease management.
